The article "Clinical Promotion of Comfort Nursing Combined with Comprehensive Nursing in the Treatment of Severe Stroke Patients with Diabetes in ICU" was retracted in 2023. Reasons: signs of a paper mill; compromised peer review; unreliable results or conclusions.

# Clinical Promotion of Comfort Nursing Combined with Comprehensive Nursing in the Treatment of Severe Stroke Patients with Diabetes in ICU

**DOI:** 10.1155/2023/1593651

**Published:** 2023-02-03

**Authors:** Haiqin Zhang, Hongmei Chu, Xiaoli Qian, Yan Zhang, Qiuping Wang

**Affiliations:** ^1^Department of Critical Care Medicine, Hai'an People's Hospital, Nantong, Jiangsu 226600, China; ^2^Nursing Department, Hai'an People's Hospital, Nantong, Jiangsu 226600, China; ^3^Department of Neurosurgery, Outpatient and Emergency Department of Wuxi Second People's Hospital, Wuxi, Jiangsu 214000, China

## Abstract

**Objective:**

To investigate the application value of comprehensive nursing combined with comfort nursing for severe stroke patients with diabetes in the intensive care unit (ICU), as well as its effect on the incidence of pressure ulcers and aspiration.

**Methods:**

Between March 2019 and March 2021, 123 severe stroke patients with diabetes who were treated at our hospital were randomly assigned to one of two groups: the control group (*n* = 61) or the study group (*n* = 62). The control group received normal care, but the research group received comprehensive nursing as well as comfort nursing. The two patient groups were compared in terms of the effects of the clinical application.

**Results:**

The two groups did not differ significantly in general data (*P* > 0.05). The shorter ICU monitoring and extubation times, the lower incidence of pressure ulcers, aspiration, and nosocomial infections, and higher self-rating anxiety scale (SAS) and self-rating depression scale (SDS) scores and a lower MOS 36-item short-form health survey (SF-36) score were all observed in the research group when compared to the control group (*P* < 0.05).

**Conclusion:**

For severe stroke patients with diabetes in the ICU, comprehensive nursing combined with comfort nursing has a promising effect, significantly, lowering the risk of pressure ulcers, aspiration, and nosocomial infections, accelerating physical recovery, enhancing mental state, and ensuring a better prognosis, deserving general clinical promotion.

## 1. Introduction

Stroke is a common cerebrovascular disease with high mortality and disability risk. The incidence of stroke has increased in recent years due to the increasing aging of the population and alterations in a dietary structure. According to reports, one of the leading causes of disease-related death in China is stroke. Stroke not only has a high incidence, recurrence, and mortality rate but also causes functional impairment in varying degrees in about three-quarters of patients, causes excruciating physical pain and mental stress in patients, and has a significant negative impact on patients' quality of life and that of their families. The most frequent type of stroke is cerebral infarction brought on by carotid and intracranial atherosclerosis [1–3].

The comorbidity of dysphagia in patients with severe stroke may result in complications such as aspiration pneumonia and acute respiratory distress syndrome due to aspiration; In addition, patients with severe strokes who are bedridden for an extended period of time have a higher risk of developing pressure ulcers, which can hamper prognostic rehabilitation and possibly pose a threat to life without proper nursing interventions [4–7]. In order to reduce the incidence of aspiration and pressure ulcers, a therapeutic treatment must incorporate effective nursing intervention. Patients with abnormal blood glucose levels may be at a higher risk of cognitive impairment due to excessive insulin levels and insulin resistance, which also greatly increases the risk of the consequences listed. As a result, this population in the clinic needs to receive additional attention.

Because of its benefits of easy operation, low-personnel quality requirements, and widespread application, the conventional nursing intervention mode is frequently used in the care of various diseases. However, the conventional nursing lacks precise, specific, and humanized nursing measures, which make it challenging to achieve high-quality symptomatic interventions and results in an undesirable clinical nursing effect. A modified version of routine care is the comprehensive nursing, which is a model of high-quality care. The comprehensive nursing, an emerging nursing paradigm in recent years, primarily ensures nursing quality by systematizing nursing processes, integrating the advantages of responsible nursing and group nursing, and enhancing nursing work initiative and independence. The comfort nursing focuses on patient's comfort and satisfaction in fundamental nursing and nursing research, with comfort as the goal of the holistic nursing process. In order to create a mature and long-lasting clinical nursing program, this study combined the two techniques to investigate the impacts of their intervention on severely diabetic stroke patients in the intensive care unit.

## 2. Scheme Design

### 2.1. Research Object

One hundred and twenty three patients with severe stroke and diabetes who were admitted to our hospital's ICU between March 2019 and March 2021 were chosen based on the aforementioned criteria.

An online web-based randomization tool (freely available at https://www.randomizer.org/) was used to conduct the randomization. The randomization procedure and assignment were managed by an independent research assistant who was not involved in the screening or evaluation of the participants to ensure allocation concealment.

In order to detect a 3-point difference between groups in a 2-sided significance test with a power of 0.8 and an alpha error level of 0.05, the original sample size calculation predicted that 60 patients in each group would be required.

Prior to the enrollment in this study, patients signed informed consent forms. The hospital Ethics Committee gave its approval to the study protocol. JN-KI20190406 is the ethics code. All procedures adhered to the ethical principles stated in the Declaration of Helsinki for clinical research.

Inclusion criteria: ① patients whose stroke diagnosis was confirmed by the brain CT and MRI; ② patients who were clinically diagnosed as diabetic; ③ patients who were at least 18 years old and had been in the hospital for more than two weeks; ④ the Glasgow Coma Scale (GCS): 8–12 points; ⑤ the water swallow test (WST)> grade III, accompanied by swallowing dysfunction; ⑥ patients and their families were fully informed about the research process and willing to participate in this study.

Exclusion criteria: ① patients who died within seven days in ICU; ② patients whose conditions were quite severe and unstable; ③ patients with gastrointestinal diseases such as esophageal reflux; ④ patients with pressure ulcers or aspiration before admission; ⑤ patients who terminated the treatment; ⑥ patients with mental disorders and cognitive dysfunctions.

### 2.2. Grouping

In accordance with the timing of their admission, the patients were divided into two groups: the control group (*n* = 61) and the research group (*n* = 62). The implementation of this research protocol was subject to review and supervision by our hospital's ethical committee.

### 2.3. Intervention Methods

Patients in the research group received comprehensive nursing combined with the comfort nursing, while patients in the control group received routine ward management, medication guidance, condition monitoring, respiratory management, nutritional support, and other ICU nursing measures. The specific measures were as follows:

1. Formulation of nursing schemes: the nursing goals and specific intervention measures were clarified after the formation of a dedicated nursing team and the evaluation of the patients' general information, state of consciousness, vital signs, mental status, family, swallowing function, language function, motor function, and ability to perform daily activities [8–11]. 2013 The nursing scheme was then appropriately and timely adjusted in response to changes in the patient's condition.
2. Ward environment: to provide the patients a comfortable and secure environment, the ward needed to be calm, organized, and well-equipped, with a temperature of 20–24°C, relative humidity of 50–60%, good ventilation, fresh air, and soft lighting.
3. Psychological intervention: many patients suffer from negative emotions such as anxiety and depression as a result of the acute attack of stroke, which necessitates the participation of comfort and encouragement in the communication with them in order to contribute to the formation of their confidence in the disease, the enhancement of the treatment coordination, and the motivation of their engagement in family and social activities.
4. Risk assessment of pressure ulcers and aspiration: the “Pressure Ulcer Risk Assessment Form” was used to evaluate the risk for the development of pressure ulcers in combination with the patient's comprehensive nutritional status, body mass, and stool control ability; The drinking water swallow test (WST) was used to estimate the risk of aspiration in patients, with a focus on high-risk patients who require a prompt treatment.
5. Skincare: patients were helped to change positions on a frequent basis, a mattress was used to alleviate skin pressure, the bedside angle was changed suitably, and the patient's skin was washed and kept dry. Regular cleaning of the skin of the perineum and anus was necessary for patients with incontinence. To guarantee that the patients have a comfortable body feeling, clothing, quilts, sheets, and other bedding should be dry and orderly [12–14].
6. Sputum suction: the patients required regular sputum suction in order to maintain smooth breathing, which rigorously adhered to aseptic operating requirements. Following the culturing of the sputum samples in the laboratory, the nursing plan was modified in accordance with the results of the sputum test [15].
7. Health education: after a thorough review of the patient's medical records, the patients and their families received health education through collective education, group education, individual conversations. The main topics covered in this health education were the basics of preventing cerebrovascular disease, rehabilitation advice, dietary recommendations, daily routines, complications, and other health information.
8. Necessary nutritional support: utilizing a variety of resources to provide patients with enough social support and urge patients' families and friends to pay them regular visits.

### 2.4. Observational Indexes

General information: the following patient characteristics were gathered for the two patient groups: age, gender, hypertension, stroke type, focal site, stroke history, Acute Physiology and Chronic Health Evaluation II (APACHE II) score, and smoking and drinking histories.

The ICU monitoring and extubation times of the two patient groups were compared and assessed.

Pressure ulcers: there are four different levels of severity. Grade I: the skin is heated, numb, swollen, and tender, and the skin has not recovered 30 minutes after the pressure is released; Grade II: there are ulcers, blisters, and no scabs, and the skin is purple-red, swollen, and rigid. Grade III: the skin blisters have ruptured, exposing a wet, red lesion that has yellow exudate; Grade IV: necrosis and blackening of the skin tissue, local eschar, and foul-smelling purulent secretions.

Aspiration: the pepsin test in the sputum specimen was positive [16].

Mental State: prior to and following the intervention, patients' psychological states were evaluated using the self-rating anxiety scale (SAS) and self-rating depression scale (SDS). Mild anxiety was defined as 50 to 59 points, moderate anxiety as 60 to 69 points, and severe anxiety as 70 to 79 points. Mild depression was defined as 53 to 62 points, moderate depression as 63 to 72 points, and severe depression as 72 points and above. The higher the score, the more severe the psychological difficulties of the patients.

Quality of life: the prognostic quality of life of patients was evaluated using the MOS 36-item short-form health survey (SF-36) scale, which has eight dimensions with a score of 100 each. The score is directly correlated with the patient's quality of life.

The incidence of nosocomial infections: the number of nosocomial infections that occurred in the two patient groups during the nursing period was counted in order to determine the incidence of nosocomial infections.

The 2013 Chinese edition of the guideline for the prevention and treatment of type 2 diabetes is used to regulate the level of glycated hemoglobin. The goal is to keep glycosylated hemoglobin below 7%.

### 2.5. Statistical Processing

SPSS22.0 was used for the data analysis in this study to determine the difference between groups, and GraphPad Prism 7 (GraphPad Software, San Diego, USA) software was used to plot the graphs. Normally distributed measurement data were expressed as the mean ± standard deviation (*n*=2(*μ*_*α*_+*μ*_*β*_)^2^*p*(1 − *p*)/*δ*^2^), and the comparison was conducted using the *t*-test, while the analysis of the count data, represented by [*n* (%)], was conducted using the *X*^2^ test. *P* < 0.05 indicated that the difference was statistically significant.

## 3. Results

### 3.1. General Information

The general features of the two patient groups, including age, stroke type, and lesion site, were the same. (*P* > 0.05).  Table 1.

### 3.2. ICU Monitoring Time and Extubation Time

ICU monitoring and extubation times took substantially less time in the study group than that in the control group (*P* < 0.05), Figure 1.

### 3.3. Pressure Ulcers

Patients in the study group experienced pressure ulcers to a lesser extent and with a lower frequency than those in the control group (*P* < 0.05), Table 2.

### 3.4. Aspiration

The research group had a much lower aspiration rate than the control group, with only 2 cases of aspiration compared to 9 in the control group (*X*^2^ = 5.0182, *P*=0.025), Figure 2.

### 3.5. Mental State

The SAS and SDS scores of the study group were significantly lower than those of the control group (*P* < 0.05), Figure 3.

### 3.6. Quality of Life

The SF-36 score of the research group was considerably higher than that of the control group (*P* < 0.05), Table 3.

### 3.7. Nosocomial Infections

There were 3 nosocomial infections in the research group compared to 11 in the control group, showing that there was a considerably lower frequency of nosocomial infections there (*P* < 0.05), Figure 4.

### 3.8. Glycosylated Hemoglobin Level

In two groups of patients with diabetes mellitus and stroke, the amount of glycosylated haemoglobin was lower than it was prior to the intervention. (*t* = 16.823/*t* = 14.441 and *P* < 0.001/*P* < 0.001). There was no significant difference between the two groups before and after the intervention, Table 4.

## 4. Discussion

Due to the severity of their condition, patients with severe stroke frequently struggle to turn over and are unable to cough effectively. Pressure ulcers and aspiration are two common complications in people with severe strokes. Particularly for patients in the acute care period of the ICU, aspiration, to which aspiration pneumonia and acute respiratory distress syndrome are secondary, may cause a huge increase in the risk of death [17–20]. Pressure ulcers are defined as the localized tissue erosion and necrosis following blood flow obstructions brought on by persistent pressure on the patient's local tissues, which causes more discomfort and delays healing. Therefore, it is believed that effective pressure ulcer and aspiration control is essential for improving the clinical outcome of treatment for severe stroke patients who also have diabetes and nursing work [21–24].

Although conventional care can offer care for patients, the care process is fixed and the care model is singular, making it difficult to meet patients' expectations for excellent care and having certain restrictions. The enhancement of the nursing effect and the improvement of the patient's prognosis are guaranteed by the comprehensive nursing, which has all-round nursing procedures as the core framework in terms of nursing responsibilities and evaluations, standardized nursing plans, patient education plans, discharge plans, nursing forms filling, and control of nursing quality, which are interlocked and coordinated as a whole. Additionally, synergistic comfort nursing emphasizes the concept of “comfort” as part of holistic nursing in order to guarantee the most comfortable and pleasant condition in the patients' psychological, physical, and social aspects or to lessen the patients' discomfort. The purpose of this study was to provide a theoretical framework for the improvement of clinical nursing programs by investigating the impact of comprehensive nursing along with the comfort nursing on the incidence of pressure ulcers and aspiration in severe stroke patients with diabetes. This investigation was conducted in order to improve the quality of care for patients with severe stroke in the ICU.

The study's findings showed that the research group experienced shorter ICU monitoring and extubation times than the control group (*P* < 0.05), which indicates that the combination of the two nursing methods is highly effective in promoting patient recovery. It might be because the combined nursing approach is more mature and humane than traditional nursing methods, ensuring a stable recovery. The results were consistent with the research results by Hughes and Lapane [25]. Moreover, the research group in this study had a significantly lower incidence of pressure ulcers, aspiration, and nosocomial infections than the control group (*P* < 0.05), suggesting the promising efficacy of the combined nursing method adopted in this study, which may be attributed to the precautionary measures for latent high-risk complications such as pressure ulcers, aspiration, and infections after early evaluation of patients' emotional changes and clarification of the nursing orientation. On the one hand, comprehensive care includes high-quality symptomatic care techniques that lower the risk of peptic ulcer complications in patients by providing them with fundamental medical services such as health education, dietary guidance, digestive system care, and medication management. On the other hand, comfort care reduces patients' fears and stress reactions through psychological care, environmental care, and positive social support, thus improving patient's resistance and recovery [26, 27].

Additionally, the results showed that as compared to the control group, the research group had higher SF-36 scores and lower SAS and SDS scores (*P* < 0.05). With a nursing concept to conduct holistic, personalized, creative, and effective nursing practices, to meet patients' needs to the fullest extent and enhance the quality of care from various angles, comprehensive nursing combined with comfort nursing places additional importance on the mental health of the patients in contrast to conventional nursing methods that only focus on physical nursing. Modern medical research also values the integration of comfort nursing with existing nursing theories. This is because comfort care combined with integrated care involves physical and psychological care; health education can help patients alleviate fear and their stress response. Psychological care can help patients who are depressed or anxious due to medication or long-term bed rest, reduce their HAMD and HAMA scores, and improve their sleep quality [28, 29].

The advantages of integrated care combined with comfort care are as follows: ① patients can receive decent rest because of its ability to intervene on the ward. ② Its capacity to monitor the situation and minimize harm. ③ It enables psychological intervention and health education, and can raise patients' awareness of comprehensive care and lessen their negative feelings. ④ It makes it possible to perform physiological interventions and raises patient comfort. ⑤ It has the ability to step in with drugs that can control their uses and prevent accidents.

Limitation of this study: ① this study has a small sample size. Future studies will increase the sample size in order to more convincingly demonstrate the impact of comprehensive nursing along with the comfort nursing on the incidence of aspiration and pressure ulcers in severe stroke patients with diabetes in ICU. ② ICU patients with severe stroke and diabetes were included as research subjects in this study with the aim of raising nursing standards and the survival rate for ICU patients. However, the patient's follow-up nursing plan is not changed, and further clinical data support is needed to examine the overall clinical nursing model for stroke patients with diabetes. ③ The nursing effect is directly impacted by the professional quality and skills of nurses. In order to ensure that nursing work is carried out effectively in clinical practice, nursing professionals must undergo extensive training in both comfort nursing and comprehensive nursing.

In conclusion, comprehensive nursing combined with the comfort nursing has a promising effect on severe stroke patients with diabetes in the ICU, significantly reducing the incidence of pressure ulcers, aspiration, and nosocomial infections, accelerating physical recovery, enhancing mental state, and providing a better prognosis, deserving general clinical promotion.

## Figures and Tables

**Figure 1:** ICU monitoring time and extubation time. Note: the abscissa represents the evaluation index, and the ordinate represents the number of days, d; the ICU monitoring time and extubation time of the control group were as follows: (4.65 ± 1.66) and (10.07 ± 3.60); the ICU monitoring time and extubation time of the research group were as follows: (2.58 ± 1.52) and (7.74 ± 2.19); ^*∗*^indicates that there is a significant difference in ICU monitoring time between the two groups of patients (*t* = 7.2147, *P* < 0.001); ^*∗∗*^indicates that there is a significant difference in the extubation time between the two groups of patients (*t* = 4.3444, *P* < 0.001).

**Figure 2:** The incidence of aspiration in the two groups of patients (%).

**Figure 3:** SAS and SDS score ($\bar{x}$ ± *s*). Note: the abscissa represents SAS and SDS, and the ordinate represents the score; the SAS and SDS scores of the control group were as follows: (54.12 ± 4.25) and (51.87 ± 3.55); the SAS and SDS scores of the research group were as follows: (47.63 ± 3.51) and (46.52 ± 4.18); ^*∗*^indicates that the SAS scores of the two groups are significantly different (*t* = 9.2405, *P* < 0.001); ^*∗∗*^indicates that the SDS scores of the two groups are significantly different (*t* = 7.6451, *P* < 0.001).

**Figure 4:** The incidence of nosocomial infections in the two groups (%).

**Table 1:** Comparison of general information of the two groups of patients.

Indexes	Control group (*n* = 61)	Research group (*n* = 62)	*X* ^2^/*t*	*P*
Age (year)	60.58 ± 6.42	59.83 ± 6.19	0.6596	0.5108
Male/female	36/25	35/27	0.0829	0.773
Hypertension	24 (39.34)	27 (43.55)	0.2239	0.636
Stroke types			0.0654	0.798
Cerebral infarction	38 (62.30)	40 (64.52)		
Cerebral hemorrhage	23 (37.70)	22 (35.48)		
Stroke history			0.0754	0.784
Yes	12 (19.67)	11 (17.74)		
No	49 (80.33)	51 (82.26)		
Focus location			0.0782	0.780
Unilateral cerebral hemisphere	27 (44.26)	29 (46.77)		
Bilateral cerebral hemispheres	26 (42.62)	24 (38.71)		
Cerebellum and brainstem	8 (13.11)	9 (14.52)		
APACHEII scores	13.49 ± 2.17	13.65 ± 3.24	0.1893	0.8502
Smoking history	25 (40.98)	24 (38.71)	0.0663	0.797
Drinking history	31 (50.82)	35 (56.45)	0.3922	0.531

**Table 2:** The incidence of pressure ulcers in the two groups [*n* (%)].

Grading	Control group (*n* = 61)	Research group (*n* = 62)	*X* ^2^	*P*
Grade I	4 (6.56)	3 (4.84)		
Grade II	4 (6.56)	2 (3.23)		
Grade III	3 (4.92)	0 (0)		
Grade IV	2 (3.28)	0 (0)		
Total	13 (21.31)	5 (8.06)	4.3191	0.038

**Table 3:** Comparison of the SF-36 scores of the two groups ($\bar{x}$ ± *s*).

Categories	Control group (*n* = 61)	Research group (*n* = 62)	*t*	*P*
General health	54.91 ± 4.62	59.85 ± 3.74	6.2559	<0.001
Bodily pain	53.28 ± 5.03	57.88 ± 4.26	5.4763	<0.001
Social functioning	52.37 ± 4.25	57.26 ± 4.32	6.3274	<0.001
Role physical	54.87 ± 2.52	60.29 ± 3.24	10.3444	<0.001
Physical functioning	55.17 ± 2.58	58.63 ± 4.75	5.0083	<0.001
Vitality	52.73 ± 4.57	57.16 ± 4.68	5.3104	<0.001
Mental health	53.22 ± 4.50	58.25 ± 3.51	6.9186	<0.001
Role emotional	53.54 ± 4.53	60.04 ± 3.51	8.9038	<0.001

**Table 4:** Comparison of the glycosylated hemoglobin level of the two groups ($\bar{x}$ ± *s*, (%)).

Group	*n*	Before intervention	After intervention	*t*	*P*
Control group	61	10.48 ± 1.06	6.95 ± 1.25	16.823	<0.001
Research group	62	10.23 ± 1.47	7.01 ± 0.96	14.441	<0.001
*t*		1.080	−0.299		
*P*		0.282	0.617		

## Data Availability

All data generated or analyzed during this study are included in this published article.
